The article "Changes in Serum CRP and PCT Levels in Patients with Acute Simple Lower Urinary Tract Infection and Evaluation of the Efficacy of Treatment with Shuangdong Capsules" was retracted in 2024. Reasons: signs of a paper mill; suspected computer-generated content; unreliable results or conclusions; concerns about the data.

# Changes in Serum CRP and PCT Levels in Patients with Acute Simple Lower Urinary Tract Infection and Evaluation of the Efficacy of Treatment with Shuangdong Capsules

**DOI:** 10.1155/2022/9750237

**Published:** 2022-08-23

**Authors:** Yachun Tang, Qun Zhou

**Affiliations:** The Affiliated Nanhua Hospital, Department of Urology, Hengyang Medical School, Universitity of South China, Hengyang 421002, Hunan, China

## Abstract

**Objective:**

The aim of this study is to investigate the changes and significance of serum C-reactive protein (CRP) and procalcitonin (PCT) levels in patients with acute simple lower urinary tract infection (ALUTI) and to analyze the efficacy of treatment with Shuangdong capsules, so as to provide a basis for the rational clinical application of drugs.

**Methods:**

92 patients with ALUTI (observation group) were randomly divided into 46 cases each in group A and group B. Group A was treated with basic anti-infective drugs, while group B was treated with Shuangdong capsules, and the duration of treatment in both groups was 14 days. The curative effect of the two groups was analyzed, and the changes in serum PCT and CRP levels were compared before and after treatment and compared with 40 healthy people in the control group.

**Results:**

The serum PCT and CRP levels, the number of urinary leukocyte count (LEU), and the number of urinary bacterial count (BACT) were significantly higher in Group A and Group B than in the healthy control group before treatment (*P* < 0.05). After treatment, the total clinical efficiency of patients in group B (97.83%) was significantly higher than that in group A (78.26%) (*P* < 0.05). The serum PCT and CRP levels, the number of urinary LEU, and the number of urinary BACT decreased in both groups after treatment compared with those before treatment, and all of them were significantly lower in group B than in group A (*P* < 0.05). The area under the curve (AUC) values of serum PCT and CRP levels for the diagnosis of acute simple lower urinary tract infection were 0.747 (95% CI 0.633–0.860) and 0.926 (95% CI 0.870∼0.982), both with high sensitivity and specificity.

**Conclusion:**

The Shuangdong capsule combined with conventional antibacterial drugs has better clinical efficacy in the treatment of acute simple lower urinary tract infection; serum CRP and PCT levels in patients with acute simple lower urinary tract infection can be used as indicators for diagnosis and efficacy determination of the infection.

## 1. Preface

Acute urinary tract infections (AUTIs) develop as a result of multiple pathogenic bacteria attacking the urinary system and are most common in women of reproductive age, and acute lower urinary tract infections (ALUTIs), as one of the two most common types of AUTI, are most common mainly in urethritis and cystitis [1, 2]. ALUTI is generally a clinical manifestation with bladder irritation signs such as urinary frequency, urinary urgency, and urinary pain and may present with typical symptoms such as pain in the pubic area, purulent urine, hematuria, or even systemic symptoms such as fever, headache, nausea, and vomiting [3]. For LUTI, not only early recognition and timely diagnosis are needed but also a rational selection of antibiotics is essential as soon as possible, which is the key to improve its prognosis and reduce the incidence of serious complications [4]. Traditional Chinese medicine has a long history in the treatment of various infectious diseases and the curative effect is accurate. Recent studies [5, 6] have shown that the combination of the Shuangdong capsule with conventional anti-infective treatment has a better alleviating effect on symptoms such as urinary frequency, urinary urgency, burning and stinging urethra, and yellow urine in acute mild to moderate simple lower urinary tract infection with damp-heat in the lower jiao and deficiency of both qi and yin, which provides a better treatment option for AUTI.

Patients with ALUTI can be complicated by bacteremia in severe cases, which increases the risk of death; therefore, it is of great clinical importance to find effective diagnostic indicators to accurately evaluate patients' infections and guide their treatment in ALUTI patients [7, 8]. Confirmation of the diagnosis of infectious diseases relies on pathogenic testing, but bacterial culture is time-consuming and not conducive to guiding the early application of antimicrobial drugs. Inflammatory indicators that are widely used clinically and have a high reference value include white blood cell count (WBC), absolute neutrophil count (ANC), C-reactive protein (CRP), and procalcitonin (PCT) [9, 10]. CRP is an acute chronotropic response protein, a nonspecific inflammatory indicator that can be elevated in bacterial infections, and PCT is a nonhormonally active glycoprotein that can be significantly elevated in systemic infections [11, 12]. Both are important biological indicators for the serological diagnosis of infectious diseases and have great clinical significance in identifying infectious diseases and assessing the severity of bacterial infections.

In this study, we selected patients with acute simple lower urinary tract infection divided into two groups, analyzed the therapeutic effect of Shuangdong capsule treatment on acute simple lower urinary tract infection by comparing the efficacy of the two groups and the changes in serum CRP and PCT levels in the two groups during the treatment, and evaluated the diagnostic value of serum CRP and PCT levels on acute simple lower urinary tract infection.

## 2. Data and Methods

### 2.1. Case Selection

#### 2.1.1. Western Medical Diagnostic Criteria

As referenced in the relevant authoritative literature [13, 14], acute simple lower urinary tract infections, which occurred in patients with normal functioning urinary tract anatomy and no comorbidities such as diabetes mellitus or immunocompromise, were cured by short-term antimicrobial therapy and usually did not affect the renal function.

Symptoms such as (1) frequency, urgency, painful urination, discomfort in the suprapubic bladder area or perineum, and burning sensation in the urethra; (2) terminal hematuria was frequently observed, and the body temperature was normal or only hypothermia; (3) pressure pain in the suprapubic bladder area on physical examination; (4) elevated WBC count on urinalysis (>7.41 WBC/ul in men and >12.47 WBC/ul in women); (5) positive culture of middle urine specimen; (6) positive urine nitrite; and (7) bacterial count >105/ml in urine. One or more of the symptoms in (1) and also in (4), with or without (2), (3), (5), (6), and (7) could be diagnosed.

#### 2.1.2. Traditional Chinese Medicine Diagnostic Criteria

Referring to the relevant authoritative literature [15], according to the characteristics of the formula and the functional principles of the Shuangdong capsule, it is proposed to select damp-heat in the lower jiao and deficiency of both qi and yin as the TCM evidence types in this study.

#### 2.1.3. Inclusion Criteria

The inclusion criteria were as follows:

1. Those who met the diagnostic criteria of Chinese and Western medicine.
2. Duration of disease <72 h.
3. Age ≥18 years.
4. Chinese medicine diagnosis of damp-heat in the lower jiao and deficiency of both qi and yin.
5. Those who did not take antifungal drugs or antibiotics within the last 3 days.
6. Those who were conscious, able to cooperate with the completion of this study, and signed the informed consent, which was reviewed and approved by the ethics committee of our hospital.

#### 2.1.4. Exclusion Criteria

The exclusion criteria were as follows:

1. The presence of urinary tract stones, urinary tract malformations, tumors, and other diseases.
2. Diagnosis of complicated urinary tract infection or upper urinary tract infection.
3. Being pregnant or in lactation.
4. Presence of abnormal cognitive, consciousness, mental, and other states.
5. Those with insufficiency of heart, liver, kidney, and other organs.
6. Allergic to drugs related to this study.
7. Combined with vaginal inflammation, genital ulcers, or gonorrhea.

### 2.2. Clinical Data

92 patients with ALUTI (observation group) attending our hospital from July 2020 to January 2021 were randomly divided into 46 cases each in group A and group B. Group A was given basic anti-infective drug treatment, and group B was treated with the Shuangdong capsule, and the duration of treatment in both groups was 7 days. 40 healthy individuals were also selected as the control group, and there was no statistically significant difference in the comparison of the general conditions of the three groups (*P* > 0.05). See Table 1.

### 2.3. Treatment Methods

In the observation group, patients in group A received basic treatment after admission, using the appropriate antibiotics (quinolones, penicillins, cephalosporins, etc.) for no more than 7 days of antibiotic treatment, and those whose symptoms and signs disappeared and whose urine leukocytes and bacterial culture were negative during the medication period; although the course of treatment was not enough for 7 days, they could stop the medication at any time and record the time to attain healing. The end follow-up was performed on day 8 to determine whether there was a relapse (relapse criteria: those with symptoms and signs recurring, along with positive urine leukocytes, or positive urine bacterial culture). Patients in group B were given Shuangdong capsules (produced by Guizhou Long-range Pharmaceutical Co., Ltd., 0.3 g/capsule), 0.9 g/dose, 3 times/day, for 7 days on top of group A.

### 2.4. Observation Indexes

#### 2.4.1. Efficacy Evaluation

The efficacy evaluation was performed in 3 aspects: symptoms and signs, routine urine examination, and bacteriological examination. Cure: subjects' symptoms and signs reached the level of cure, urine routine and white blood cells returned to normal, and there was a negative bacterial culture at the return visit on the 8th day after the end of 7 days of drug administration. Improvement: clinical symptoms and signs were significantly improved, and 2 consecutive bacteriological examinations at different time periods converged to the normal value range, but the relevant laboratory examination indexes were partially and completely restored. Ineffective: subjects were clinically ineffective (no significant relief, persistent signs and symptoms of infection, or recurrence of signs and symptoms at or before the day 8 visit after 7 days of dosing), not cleared of bacteria, elevated urine leukocytes, or all three at the end of the 7-day visit. If one of the subject's clinical signs and symptoms and bacteriological findings were invalid and the other was missing, it was determined to be ineffective.

#### 2.4.2. Serum CRP, PCT Assay, and Urine Biochemical Indexes

The PCT level was measured before treatment by using the Ultimate semi-automatic quantitative analyzer (Shenzhen Mindray Biomedical Electronics Co., Ltd.) with the microimmunofluorescence method, and the CRP level was measured before treatment by using the automatic specific protein analyzer (Beckman Array, USA) with the rate scattering turbidimetric method, and each index was measured by the same method after treatment. The urine biochemical indicators included urine leukocyte count (LEU) and urine bacterial count (BACT), and the specimens were all midstream urine.

### 2.5. Statistical Methods

SPSS22.0 statistical software was applied. The mean, standard deviation, and percentage were used for statistical description; one-way variance (F), *t* test, or *χ*^2^ test were used to compare the serum CRP, PCT, and urine biochemical indexes and the western clinical efficacy of patients before and after treatment. The receiver operating characteristic curve (ROC) and the area under the curve (AUC) were used to judge the diagnostic efficacy of PCT and CRP. *P* < 0.05 was considered a statistically significant difference.

## 3. Results

### 3.1. Comparison of Clinical Data of the Three Groups

The clinical data of the three groups were compared, and the results showed that the comparison of gender, age, height, weight, proportion of smoking, and the proportion of alcohol consumption in the control group, group A, and group B indicated no statistically significant differences (*P* > 0.05); no statistically significant differences were found between group A and group B in terms of disease duration, proportion of initial disease onset, and the proportion of recurrence (*P* > 0.05). Table 1.

### 3.2. Comparison of Serum and Urine Indexes before Treatment in the Three Groups

The data of serum indexes and urinary biochemical indexes of diseased patients and healthy individuals were compared, and the results showed that the serum CRP, PCT level, number of urinary LEU, and number of urinary BACT in the healthy control group were significantly lower than those in group A and group B (*P* < 0.05); the differences between serum CRP, PCT level, number of urinary LEU, and number of urinary BACT before treatment in group A and group B were not statistically significant (*P* > 0.05). See Figure 1.

### 3.3. Clinical Efficacy of Group A and Group B

The proportion of cured, improved, and invalid patients in group A was 34.78%, 43.48%, and 21.74%, respectively, and the total effective rate was 78.26%. The proportion of cured, improved, and invalid patients in group B was 65.55%, 43.48%, and 21.74%, respectively, and the total effective rate was 97.83%. A comparison of the total effective rate between group A and group B showed that group B was significantly higher than group A (*P* < 0.05). See Table 2.

### 3.4. Comparison of Serum and Urine Indexes between Group A and Group B after Treatment

Comparing the data of serum indexes and urinary biochemical indexes between group A and group B after treatment, it could be found that the two treatment regimens had different degrees of influence on the levels of serum CRP and PCT, the number of urinary LEU, and the number of urinary BACT in patients with acute simple lower urinary tract infection, and all of them could reduce the levels of serum inflammatory factors and urinary biochemical indexes, but the reduction was more significant in group B with the combined application of the Shuangdong capsule (*P* < 0.05).  Figure 2.

### 3.5. Analysis of the Value of Serum CRP and PCT Levels for the Diagnosis of Acute Simple Lower Urinary Tract Infection

The AUCs of serum CRP and PCT levels for the diagnosis of acute simple lower urinary tract infection were 0.747 (95% CI 0.633–0.860) and 0.926 (95% 0.870–0.982), respectively. Among them, PCT had the highest diagnostic value for acute simple lower urinary tract infection, with a sensitivity of 80.40% and specificity of 95.00% when the optimal cutoff value was 0.754. See Table 3 and Figure 3.

## 4. Discussion

ALUTI is a common and frequent clinical disease with a high incidence, and patients often present with symptoms such as urinary frequency, urinary urgency, and painful urination; in severe cases, symptoms of systemic infection may occur, requiring reasonable antimicrobial therapy with antibacterial drugs [16]. Clinically, different antibacterial drugs are often taken for the treatment of different pathogenic bacteria, and among the treatments for UTI, antibiotics are definitely effective, but before the results of urine bacterial culture drug sensitivity are obtained, drugs can only be used based on clinical experience, which sometimes delays the treatment and prolongs the treatment time [17, 18]. Inflammation caused by LUTI stimulates local leukocytes or platelets to trigger coagulation, leading to the production of vasoactive chemokines and cytokines as well as triggering an increase in the synthesis of serum CRP, making serum CRP a useful indicator for detecting infection [19]. Serum CRP levels can play a positive role in the diagnosis and prognosis of infectious diseases, which is consistent with the results of this study.

In recent years, many herbs that clear heat and detoxify toxins and dampness have been shown to have inhibitory effects on pathogenic microorganisms and can inhibit or destroy the formation of toxic substances. Acute simple lower urinary tract infection belongs to the category of “hot lung” in ancestral medicine, and its pathogenesis is the accumulation of dampness and heat in the lower jiao and unfavorable qi-transformation in the kidney and bladder. While the Shuangdong capsule is composed of *Gardenia jasminoides*, *Astragalus membranaceus*, *Oldenlandia diffusa*, lilyturf root, bitter wood, and cluster mallow fruit, which has the effect of clearing heat and clearing lung, benefiting qi and nourishing yin, and can better relieve symptoms such as urinary frequency, urinary urgency, burning and stinging pain in the urethra, and yellow urine [20] Therefore, in this study, some patients were treated with the Shuangdong capsule in addition to conventional antibacterial therapy. The results showed that the clinical efficacy and improvement of urinary biochemical indexes of patients in group B treated with the Shuangdong capsule were significantly better than those in group A treated with conventional antibacterial therapy. Comparing patients with acute simple lower urinary tract infection with healthy physical examiners, we were able to find that serum CRP and PCT levels increased in patients after acute simple lower urinary tract infection, while serum CRP and PCT levels responded differently to the effects of different treatment regimens, and under the effect of therapeutic drugs, serum CRP and PCT levels in both group A and group B decreased compared with those before treatment, and the decrease in group B was significantly greater than that in group A. Analyzing the reasons for this, the Shuangdong capsule has the function of clearing heat and promoting lymphatic flow, benefiting qi and nourishing yin, and it can be used in combination with antibacterial drugs to treat both the symptoms and signs of patients, as well as potentially enhance the immunity of the body, which can obtain better efficacy and improve the rational use of drugs [21, 22].

ALUTI is a common clinical inflammatory disease that requires timely and effective treatment, and the prerequisite for such treatment is an accurate diagnosis. The current “gold standard” for clinical diagnosis of ALUTI is a urine midstream culture, which takes a long time and is influenced by the sample taken from the patient, so other tests are needed. The biomarker procalcitonin (PCT) has been shown to be a good diagnostic indicator for predicting bacterial infections such as sepsis and pneumonia, thereby reducing unnecessary antibiotic exposure [23, 24]. PCT provides additional benefits in guiding antibiotic therapy in UTI patients compared to other biomarkers. CRP is an acute timing reactive protein secreted by liver cells and is one of the indicators for early diagnosis of inflammation [25]. When the body is affected by a bacterial or fungal infection or tissue damage, its level can be rapidly increased and can be rapidly decreased when the disease recovers. In this study, CRP and PCT had a certain diagnostic value for acute simple lower urinary tract infection, and the levels of PCT and CRP in serum decreased with the gradual improvement of the disease in both groups, suggesting that the levels of PCT and CRP in serum can be used as an auxiliary parameter to judge the efficacy and prognosis of ALUTI.

In conclusion, the Shuangdong capsule combined with conventional antibacterial drugs for the treatment of acute simple lower urinary tract infection has better clinical efficacy, and different treatment regimens for patients with different efficacy values also caused different changes in CRP and PCT levels. These changes can be more accurate and sensitive to determine the patient's condition, that is, CRP and PCT levels can be used as indicators for the diagnosis and efficacy of acute simple lower urinary tract infection.

## Figures and Tables

**Figure 1:** Comparison of serum and urine indexes before treatment in the three groups. Contents in (a–d) are CRP, PCT, LEU, and BACT, respectively. ▲*P* < 0.05 compared with the control group.

**Figure 2:** Comparison of serum and urine indexes between group A and group B after treatment. Contents in (a–d) are CRP, PCT, LEU, and BACT, respectively. ▽*P* < 0.05 compared with group A.

**Figure 3:** ROC curve of the diagnostic value of serum CRP and PCT levels for acute simple lower urinary tract infection.

**Table 1:** Comparison of clinical data of the three groups (*n*, Mean ± SD).

Indicator		Control group (*n* = 40)	Group A (*n* = 46)	Group B (*n* = 46)	*F/t/χ * ^2^ value	*P* Value
*Gender (%)*	Male	6 (15.00)	7 (15.22)	6 (13.04)	0.105	0.949
	Female	34 (85.00)	39 (84.78)	40 (86.96)		
Age (years)		45.26 ± 4.28	46.36 ± 4.13	47.06 ± 3.89	2.087	0.129
Height (m)		1.62 ± 0.08	1.61 ± 0.12	1.62 ± 0.10	0.143	0.867
Body weight (kg)		60.40 ± 6.25	59.80 ± 7.10	60.64 ± 7.23	0.180	0.836
Duration of illness (h)		—	36.38 ± 10.12	37.24 ± 9.87	0.269	0.789
Smoking (%)		8 (20.00)	10 (21.74)	9 (19.57)	0.074	0.964
Drinking alcohol (%)		7 (17.50)	8 (17.39)	6 (13.04)	0.434	0.805
First attack (%)		—	25 (54.35)	22 (47.83)	0.392	0.532
Relapse (%)		—	21 (45.65)	24 (52.17)		

**Table 2:** Clinical efficacy of group A and group B (*n*, %).

Group/Effectiveness	Group a (*n* = 46)	Group B (*n* = 46)	*χ * ^*2*^ value	*P* Value
Cure	16 (34.78)	30 (65.55)	—	—
Improvement	20 (43.48)	15 (32.61)	—	—
Ineffective	10 (21.74)	1 (2.17)	—	—
Total effective rate	36 (78.26)	45 (97.83)	8.364	0.004

**Table 3:** Analysis of the value of serum CRP and PCT levels for the diagnosis of acute simple lower urinary tract infection.

Indicator	AUC	95% CI	Best cutoff value	Sensitivity (%)	Specificity (%)
CRP	0.747	0.633∼0.860	0.584	60.90	97.50
PCT	0.926	0.870∼0.982	0.754	80.40	95.00

## Data Availability

The data involved in this trial were obtained from the authors through reasonable requests to the corresponding author.
